RETRACTED

# Exosomal miR-27b-3p Derived from Hypoxic Cardiac Microvascular Endothelial Cells Alleviates Rat Myocardial Ischemia/Reperfusion Injury through Inhibiting Oxidative Stress-Induced Pyroptosis via Foxo1/GSDMD Signaling

**DOI:** 10.1155/2022/8215842

**Published:** 2022-07-06

**Authors:** Baojian Zhang, Chao Sun, Yaozhong Liu, Fan Bai, Tao Tu, Qiming Liu

**Affiliations:** ^1^Cardiac Care Unit, Affiliated Hospital of Traditional Chinese Medicine, Xinjiang Medical University, Urumqi City, Xinjiang Uygur Autonomous Region, China; ^2^Department of Cardiology/Cardiac Catheterization Lab, Second Xiangya Hospital, Central South University, Changsha, Hunan, China

## Abstract

**Background:**

Exosomes derived from cardiac microvascular endothelial cells (CMECs) under hypoxia can mediate cardiac repair functions and alleviate pyroptosis and oxidative stress during ischemia-reperfusion (I/R) injury. This study is aimed at investigating the effect and mechanism of miR-27b-3p underlying hypoxic CMECs-derived exosomes against I/R injury.

**Methods:**

CMECs were isolated from the left ventricle of Sprague-Dawley rats, followed by culturing under hypoxic conditions or pretreatment with the miR-27b-3p inhibitor. CMECs-derived exosomes were added into H9C2 cells before hypoxia/reoxygenation (H/R) or injected into the rat heart before I/R injury. An *in vivo* I/R injury model was established by ligating and releasing the left anterior descending coronary artery. Expression of pyroptosis-related factors was detected using Western blot, and heart infarcted size was determined by the 2,3,5-triphenyl-2H-tetrazpinolium chloride staining method. Dual-Luciferase Reporter assays were performed to analyze the interactions of nmiR-27b-3p-forkhead box O1 (Foxo1) and Gasdermin D- (GSDMD-) Foxo1. Chromatin-immunoprecipitation (ChIP) assays were performed to validate the interactions between forkhead box O1 (Foxo1) and Gasdermin D (GSDMD) and Foxo1-mediated histone acetylation of GSDMD.

**Results:**

CMECs were successfully identified from left ventricle of Sprague-Dawley rats. The expressions of Foxo1 and pyroptosis-related proteins (GSDMD, NLPR3, cleaved caspase 1, IL-1*β,* and IL-18) were upregulated in the rat heart after I/R injury. Treatment of CMEC-derived exosomes, especially that under hypoxic conditions, significantly reduced pyroptosis in the rat heart. miR-27b-3p was significantly upregulated in CMEC-derived exosomes under hypoxic conditions, and miR-27b-3p inhibition in exosomes alleviated its cytoprotection and inhibited oxidative stress in H9C2 cells. Treatment with Foxo1 overexpression plasmids aggravated *in vitro* H/R and *in vivo* I/R injury by upregulating pyroptosis-related proteins. Further experiments validated that miR-27b-3p negatively targeted Foxo1, which bound to the promoter region of GSDMD.

RETRACTED

**Conclusions:**

These results demonstrated a great therapeutic efficacy of miR-27b-3p overexpression in hypoxic CMEC-derived exosomes in preventing the development of myocardial damage post I/R injury through inhibiting Foxo1/GSDMD signaling-induced oxidative stress and pyroptosis.

## 1. Introduction

Myocardial infarction (MI), a life-threatening disease worldwide, is the most common in Europe and the United States. Annually, there are about 1.5 million myocardial infarction in the United States. In recent years, China has shown an obvious increasing trend, with at least 500000 new cases per year and at least 2 million current cases. The most commonly used treatment for MI in clinical practice is reperfusion therapy, which causes myocardial ischemia-reperfusion (I/R) injury to produce irreversible damage to cardiomyocytes and myocardial diastolic dysfunction [1]. Therapeutic reperfusion could result in complications through initiating multiple pathophysiological processes, including myocyte necrosis, microvascular obstruction, and microcirculation dysfunction [2–4].

Cardiac microvascular endothelial cells (CMECs) are important cells in the myocardium. Abnormal and detrimental changes in CMECs in responses to I/R include excessive inflammation, apoptosis, and reactive oxygen species (ROS) production, which could contribute to the progression of cardiac dysfunction [2, 4–6]. CMECs constitute the microcirculatory tract and play crucial roles in causing cardiac microvasculature injury in I/R [2, 4]. CMECs secrete a wide range of cytokines, cellular contents, and exosomes that mediate functional interactions between cardiomyocytes, leukocytes, and the circulation [2, 4, 7, 8]. Accordingly, CMECs are commonly used to mimic actual pathological state and I/R injury and have been applied in *in vitro* drug research [6]. NLRP3 inflammasome-induced pyroptosis in CMECs under I/R injury aggravates I/R-induced damage [9, 10]. Under I/R conditions, NLRP3 inflammasome is induced to stimulate caspase-1 cascade, which is responsible for the upregulation of cytokines (including interleukin- (IL-) 1*β* and IL-18) and the activation of caspase-11/gasdermin-D (GSDMD) cascade [4, 11]. Recent studies showed that exosomes derived from endothelial cells (ECs) and mesenchymal stem cells (MSCs) mediate strong cardiac repair functions of cardiomyocytes, smooth muscle cells, and fibroblasts as well as protecting against NLRP3 inflammasome-induced pyroptosis [11–16].

Exosomes are nanosized and lipid-bilayer-enclosed extracellular vesicles released by all cells that circulate in the blood. Exosomes contain RNA, lipids, and proteins and deliver signals to target cells, which is essential for intercellular communication and exchange of genetic information [17]. Exosomes derived from stem cells could inhibit inflammation and doxorubicin-induced pyroptosis in cardiac cells [11, 18, 19]. Dargani et al. [18] indicated that doxorubicin promotes the expression of IL-1*β* and IL-18 in exosomes derived from embryonic stem cells. Evidence showed that the abundance of exosomal proteins, mRNA, and miRNA and exosomal therapeutic potential could be enhanced by hypoxia [20–23]. Hypoxia stimulates the expression of miRNAs (including miR-27b-3p, miR-17-1-3p, and miR-217-3p) and proteins in cardiomyocyte or CPC-derived exosomes with cytoprotection, proangiogenic, and antifibrotic effects [20, 22, 24, 25]. However, no studies demonstrated that exosomal-derived miRNAs can protect against damage caused by I/R models; therefore, this study treated I/R model rats with CMEC-derived exosomes to explore the role of CMEC-derived exosomes in I/R model rats. Also, less was known on the effect of hypoxic CMEC-derived exosomes on I/R injury.

RETRACTED

Here, in our study, we demonstrated the protective effect of miR-27b-3p on CMEC-derived exosomes against I/R injury. Furthermore, hypoxia treatment increased exosomal miR-27b-3p and showed a higher efficacy in alleviating I/R-induced infarction size and myocardial damage in the rat heart. The mechanism of miR-27b-3p-forkhead box O1 (Foxo1) in inflammation-induced pyroptosis in the progression of I/R injury was explored in the *in vitro* and *in vivo* rat model of I/R injury. These data confirmed the myocardial protective potential of using CMEC-derived exosomes under hypoxic conditions.

## 2. Materials and Methods

### 2.1. CMEC Isolation, Identification, and Culture Conditions

The results of the isolation and identification of CMEC cells were provided by Wuhan Procell Life Sci&Tech Co., Ltd. Rat CMECs were dissociated from the left ventricle of Sprague-Dawley rats (3-4 weeks old; Disease Control and Prevention Center of Hubei, Wuhan, China) as previously described [26]. In brief, the left ventricle was isolated, minced into pieces (1 mm^3^), washed in PBS (containing 1% penicillin-streptomycin; Procell, Wuhan, China; PB180120), and digested in 0.1% trypsin (Procell, PB180225). The cells were filtrated and centrifuged at 300 × g for 5 minutes (min), followed by incubation in complete CMEC medium (Procell, CM-R135) containing 10% fetal bovine serum (FBS; Hyclone; cat. no. 10099-141) and 1% penicillin-streptomycin at 37°C with 95% air plus 5% CO_2_. The medium was replaced medium every three days. The expression of CD31 in CMECs was detected using immunofluorescence assay.

RETRACTED

### 2.2. Clinical Sample Collection

We collected the blood samples from 32 clinical patients, including 16 nonmyocardial infarction patients and 16 patients with myocardial infarction (11 women and 21 men aged 12-80 years) and took the mRNA from patient plasma to study the expression of miR-27b-3p in patients with myocardial infarction and nonmyocardial infarction.

### 2.3. Cell Transfection and Treatment

miR-27b-3p inhibitor was purchased from GenePharma (Shanghai, China) and used in cellular transfections according to the manufacturer's recommendation. miRNA inhibitor as a chemically modified RNA single strand can competitively bind with mature miRNA sequence. Moreover, it can specifically target and knock out a single miRNA molecule, weaken the gene silencing effect of endogenous miRNA, improve protein expression, conduct loss of function research, and be used to screen miRNA target sites. 1.0 × 10^5^ CMECs were placed into 6-well plates filled with fresh complete medium containing Umibio®Exosome-Free FBS medium (Umibio, Shanghai, China; cat# UR50202) and maintained for 12 hours (h) to reach 80% confluence. Then, the cells were treated with 50 nmol miR-27b-3p or NC inhibitors using Lipofectamine 2000 (Invitrogen, California, USA) for 48 h in triplicate. For hypoxia treatment, the cells were maintained in complete medium in triplicate at 37°C with 5% CO_2_ and 95% N_2_ (hypoxic conditions) for 12 h in a trigas incubator (HF100, HealForce, Hong Kong).

### 2.4. Isolation and Identification of Exosomes

The isolation of CMEC-derived exosomes was conducted using total exosome-isolation kit (Thermo Fisher, USA), according to the manufacturer's instructions. The treated cell culture was harvested by centrifugation (3000 rpm at 4°C for 15 min; 15,000 × g for 30 min) twice to remove microvesicles. After filtration (0.22 *μ*m), the exosomes were pelleted twice (100,000 × g, 4°C for 1 h; centrifuged at 120,000 × g, 4°C for 1 h) and then suspended in PBS. Exosome morphology was detected under a transmission electron microscopy (TEM, 120,000x; FEI Tecnai G12, Philips, Netherlands). The size of exosome was measured using NanoSight NS300 nanoparticle tracking analysis (Malvern, UK). Exosomal protein quantification was determined using the BCA methods (Thermo Scientific; Waltham, MA, USA; Cat #23227). The expression of exosomal markers CD63, CD81, and TSG101 were detected in triplicate by Western blotting analysis.

### 2.5. H9C2 Cell Culture, Transfection, and Treatments

The rat origin H9C2 cell line was obtained from ATCC (Manassas, VA, USA) and incubated in high-glucose DMEM (Hyclone, USA; Cat.No.SH30022.01B) containing FBS (Hyclone) and 1% penicillin-streptomycin at 37°C with 95% air and 5% CO_2_. The Foxo1 expressing pcDNA vector (Vipotion, Guangzhou, China) was constructed into *Eco*RI/*Bam*HI sites of pcDNA 3.0 vector. A total of 1.0 × 10^5^ H9C2 cells were placed into 6-well plates to 80% confluence, and the cells were treated with 4.0 *μ*g Foxo1 plasmids using Lipofectamine 2000.

RETRACTED

For the construction of cellular hypoxia/reoxygenation (H/R) model, transfected H9C2 cells were incubated under 2 h hypoxic (5% CO_2_ and 95% N_2_) plus 4 h normal conditions (H/R condition) at 37°C. Then, the H9C2 cells were incubated in medium supplemented with 50 *μ*g/ml exosomes isolated from CMECs with or without miR-27b-3p inhibitor under hypoxic conditions for 48 h.

### 2.6. Cell Proliferation Analysis

For the cell viability assay, the transfected H9C2 cells (1.0 × 10^5^/ml) were plated into 96-well plate overnight. 50 *μ*g/ml exosomes after subjecting to H/R were added into the plates and incubated for 24, 48, and 72 h. Then, the cells were incubated in CCK8 working solution (10 *μ*l, 5 mg/ml; Beyotime, Shanghai, China) in the dark for 1 h. The absorbance at 450 nm was recorded using a microplate reader (BioTek Instruments, Winooski, VT, USA).

### 2.7. I/R Model Construction and Intervention

Research approval was obtained from the Ethical Committee of Animal Experimentation of the Second Xiangya Hospital, Central South University. Healthy male Wistar rats (300 g-350 g) were randomly assigned into three sections. Forty-eight rats in the first part were grouped into four groups according to the surgery and treatment strategy (*n* = 12). Rats in the I/R model group received I/R surgery. All the animals were anesthetized with pentobarbital sodium (50 mg/kg) via intraperitoneal injection. After disinfection, the heart was exposed. The left coronary artery was ligated for 30 min and released to allow blood reperfusion for 120 min. Before I/R surgery, 12 rats were administrated with exosomes (10 *μ*l, 6 × 10^12^ particles; intramyocardial injection) derived from CMECs cultured under normal and hypoxic conditions, respectively. Rats in the control group (*n* = 12) received sham operation without ligation or reperfusion. Forty-eight rats in the second part were treated with I/R and then injected (intramyocardial injection) with 20 *μ*l lentivirus plasmid carrying Foxo1 (*n* = 24; 1 × 10^8^ TU/ml) or lentivirus vector (negative control (NC); *n* = 24) and given with free access to water and food. Forty-eight rats in the third part were injected (intramyocardial injection) with 20 *μ*l lentivirus plasmid carrying Foxo1 (*n* = 24; 1 × 10^8^ TU/ml) or lentivirus vector (negative control (NC); *n* = 24) and then treated with I/R. The lentivirus-containing Foxo1 and empty vector were purchased from GenePharma. After 7 days, intramyocardial injection with exosome isolated from CMECs was performed on all the rats. Immediately after 2 h reperfusion, the blood sample was collected from femoral arteries of each rat. Then, all rats were sacrificed using a Quietek CO_2_ Delivery Systems (Electron Microscopy Sciences), and the rat hearts were isolated and prepared for the examination of infarcted volume, histological examination, Western blot, and PCR analysis.

RETRACTED

### 2.8. Enzyme-Linked Immunosorbent Assay (ELISA)

The rat blood serum and the supernatant of H9C2 cells were prepared and used for the examination of creatine kinase (CK). Lactate dehydrogenase (LDH; Nanjing Jiancheng Biological Engineering Institute, Nanjing, China; Cat# A020-2), interleukin (IL)-1*β* (Elabscience, Wuhan, China; Cat# E-EL-R0012c), and IL-18 (Elabscience; Cat# E-EL-R0567c) were detected using the commercial ELISA kits, according to the manufacturer's recommendation.

### 2.9. ROS and SOD Detection in H9C2 Cells

The level of intracellular ROS was detected using 2′,7′-dichlorofluorescin diacetate (DCFH-DA, D6883, Shanghai, Sigma). Cells were harvested after treated with hypoxia/reoxygenation and exosomes and were incubated with 5 *μ*M DCFH-DA for 30 min at 37°C in the dark, and then, DCF fluorescence was assayed using the microplate reader (Biotek, USA) at excitation (488 nm) and emission (525 nm) wavelengths. The SOD in H9C2 cell culture supernatant was detected by SOD kits (BC0170, Solarbio Science and Technology Co., Ltd., Beijing.). After the H9C2 cells were treated with hypoxia/reoxygenation and exosomes, the supernatant of H9C2 cells was collected and tested for SOD by SOD kits. The procedure and result analysis of SOD assays refer to the instruction of SOD kits.

### 2.10. Lesion Volume Determination

The heart was quickly removed, cleaned and squeezed, dipped in dry blood, and rinsed in 4°C normal saline, followed by dipping the heart in dry and freezing in the refrigerator at -20°C for 15 min until the heart hardened. Next, the heart was taken to be cut into 1 mm thick slices using a blade from the apex to the bottom of the heart along the direction of atrioventricular sulcus. Five slices in total was prepared, and then, the slices were quickly placed in 5 ml 37°C 1% in TTC phosphate buffer (Guduo, Shanghai, China) at pH 7.4. The infarct area was white, the infarct border area was brick red, and the normal area was red. The slices were photographed using a camera.

### 2.11. Immunofluorescence Assay

PKH67 labeling of exosomes and exosomal uptake into H9C2 cells was performed as previously reported [27]. Cellular slides were fixed in 4% paraformaldehyde for 15 min and incubated with 5% Triton X-100 in PBS for 20 min, blocked with goat serum (Boster, Wuhan, China) for 30 at room temperature, with F-actin (1: 100; ab205, Abcam, Cambridge, MA, USA) at 4°C overnight, with secondary antibody (Cy3-labbeled goat-anti-rabbit IgG; Boster; BA1032) at 37°C for 1 h. DAPI was used for nuclear staining. The cells were also labeled with lipid membrane dye PKH76 (Sigma-Aldrich). An Olympus microscope (Olympus, BX53, Tokyo, Japan) was used for the capturing cellular images.

RETRACTED

### 2.12. Histological and Immunochemistry Examination

The hearts were fixed (10% formaldehyde; Beyotime), dehydrated, paraffin-embedded, and sectioned (4 *μ*m thick) using a microtome (Leica, Nussloch, Germany). Hematoxylin and eosin (HE) staining (Sigma) was performed on tissue slices according to previously reported methods [28]. For immunochemistry analysis of caspase-1, the sections were pretreated in H_2_O_2_ solutions, blocked by goat serum (Boster), and incubated with primary antibody against caspase-1 (1: 50; ab74279, Abcam,) at 4°C overnight. Secondary incubation was conducted using goat anti-rabbit IgG (1 : 1000, Abcam) in the dark for 2 h. The slices were then treated in DAB solution and Harris' hematoxylin. A BX-51 light microscopy (Olympus, Japan) was used for photographing (magnification ×200 and ×400).

### 2.13. Western Blot Analysis

The protein samples were isolated from the exosomes, rat hearts, or H9C2 cells using lysis buffer (Beyotime). The protein lysates were quantified using Bradford protein assay kit (Thermo Fisher Scientific Inc.), followed by protein separation on SDS-PAGE (10%; Beyotime) and transferring onto PVDF membranes (Millipore, Billerica, MA, USA) according to the standard methods. The expression of CD63 (1 : 1000, GTX37555, GeneTex), CD81 (1 : 500, ab109201), TSG101 (1 : 500, ab125011), Foxo1 (1 : 1000, ab39670), GSDMD (1 : 1000, ab219800), NOD-like receptor protein 3 (NLRP3; 1 : 1000, ab263899), caspase-1 (1 : 1000, ab286125) proteins, and GAPDH (1 : 10000, ab8245) were detected using specific primary antibodies at 4°C overnight. The primary antibodies were purchased from Abcam. Secondary incubation was conducted using HRP goat anti-rabbit/mouse IgG antibodies (Boster; 1 : 20000). GAPDH was used as the reference protein. The integral optical density values of proteins were analyzed using Image-Pro Plus 6.0 software.

### 2.14. Reverse Transcription Quantitative PCR (RT-qPCR)

Total RNA was extracted from the treated exsomoses, cells, or fresh heart tissues using TRIzol according to the manufacturers' instruction (Invitrogen). RNA was reversely transcribed to cDNA templates using 5x primeScript RT Master MIXperfect (TAKARA, Japan). RT-qPCR reaction was performed using Power SYBR Green PCR Master Mix (Thermo Fisher, Germany) using synthesized primers (Table 1). PCR amplification reaction conditions were at 95°C for 4 min, 40 cycles at 95°C for 20s, at 60°C for 30 s, and at 72°C for 30 s. The 2^-△△ct^ method was used for calculating the relative expression levels of gene. GAPDH and U6 served as the reference internal gene for mRNA and miRNA, respectively.

RETRACTED

### 2.15. Luciferase Reporter Assay

The interaction between miR-27b-3p and Foxo1 target was predicted using TargetScan Human (http://www.targetscan.org/vert_71/) and was validated using the dual-luciferase reporter assay [29]. The interaction between GSDMD and Foxo1 was predicated using JASPAR database (http://jaspar.binf.ku.dk/) (updated 2020) [30]. The luciferase vectors containing wild-type and mutant 3′UTR reporters of Foxo1, and the dual-luciferase reporter gene vectors of GSDMD promoter carrying the wild-type binding sites of Foxo1 were purchased from Vipotion (Guangzhou, China) and used for dual-luciferase reporter assay. miR-27b-3p mimics and negative control mimics were purchased from GenePharma and used with Lipofectamine 2000 for cellular transfections. The relative fluorescence intensities were detected 48 h after the cell transfection according to the manufacture's instruction of luciferase reporting system (Promega, Mannheim, Germany).

### 2.16. Methylation-Specific PCR (MSP) Assay

The effect of miR-27b-3p expression on the promoter methylation level of GSDMD gene was detected using MSP analysis. In brief, the H9C2 cells (1 × 10^5^) were transfected with 50 nmol inhibitor and mimics for 48 h. Cellular DNA was isolated and then sodium bisulfite-modified using EpiTect Bisulfite Kit (Qiagen, CA, USA). The samples were then desulfonated and purified and used for the measurement of methylation level using MSP. The primer sequences for amplifying GSDMD promoter region (between -1700 bp and -2100 bp) are listed in Table 1. PCR was conducted using Phanta® Uc Super-Fidelity DNA Polymerase (1 U/*μ*l; Novozyme Company, Novonordisk, Denmark) under the following reaction conditions: at 95°C for 3 min, 40 cycles of 95°C for 15 seconds (s), at 60°C for 15 s, at 72°C for 30 s, and at 72°C for 5 min. The PCR product was detected using 2% agarose gel.

### 2.17. Chromatin-Immunoprecipitation (ChIP)

ChIP assay coupled with quantitative PCR (ChIP-qPCR) was conducted to confirm the DNA-binding ability of Foxo1, HDAC2, or H3K9AC protein with GSDMD gene using a Simple ChIP Plus Enzymatic Chromatin IP Kit (CST) according to the manufacturer's protocol. The H9C2 cells were treated with protease inhibitor cocktail coupled with gradually decreased formaldehyde (37% ~1.5%) for 20 min and then blocked by glycine solution for 5 min at room temperature. Cross-linked chromatins were broken into DNA fragments using DNA micrococcal nuclease at 37°C for 20 min. ChIP reaction was conducted using 5 *μ*g of antibody against Foxo1 (1 : 30, ab39670, Abcam), H3K9AC (ab32117, 20 *μ*g/ml), HDAC2 (1 : 60, ab32117), or 1-2 *μ*l IgG (negative control) enriched in protein G magnetic beads (Invitrogen) at 4°C overnight. The immunoprecipitated complexes were then eluted using ChIP elution buffer at 65°C for 30 min, and DNA were decross-linked from proteins using proteinase K (Cell Signaling Technology) at 65°C for 2 h. The products were used for PCR of GSDMD gene using the primer pairs listed in Table 1. PrimeSTAR® HS DNA Polymerase (Takara) and a SYBR Green qPCR SuperMix kit (DBI Bioscience, Shanghai, China) were employed for PCR amplification. The DNA samples obtained were purified and subjected to PCR analysis and 2% agarose gel (Biowest, Nuaillé, France). All the reactions were performed in triplicate.

RETRACTED

### 2.18. Statistical Analyses

All the data were expressed as mean ± standard deviation. Statistical analysis was performed using GraphPad Prism 8.0 (San Diego, CA, USA). Unpaired *t*-test or one-way ANOVA followed by Tukey's post hoc test was used to analyze differences between two groups and among more than three groups, respectively. Difference at *p* < 0.05 was considered as statistically significant.

## 3. Results

### 3.1. Isolation and Identification of CMEC and Exosomes

The isolated CMECs from the rat left ventricle were CD31-positive with a purity of >90% (SupplementaryFigure 1). TEM images showed exosomes isolated from CMEC under normal and hypoxic conditions were of the expected structure and size ranging from 50 to approximately 150 nm (Figure 1(a)). NanoSight NTA showed that hypoxic conditions induced a fraction of exosomes in a range of 200~300 nm (Figure 1(b)). Western blot analysis validated high expressions of exosomal biomarkers (CD63, CD81, and TSG101 proteins) in the isolated vesicles (Figure 1(c)).

### 3.2. Hypoxic CMEC-Derived Exosomes Prevent I/R Injury and Pyroptosis and Increases miR-27b-3p Expression

To investigate the effect of hypoxic CMEC-derived exosomes on I/R injury, we injected exosomes into the heart of rats before I/R surgery. Significant MI area in the rat heart in the I/R group was seen (Figure 2(a)). The pretreatment with CMEC-derived exosomes (normal and hypoxic conditions) significantly reduced infarct area (Figure 2(a)). Western blot confirmed that the expression of Foxo1, GSDMD, NLRP3, and caspase-1 proteins were upregulated in peri-infarct tissues after I/R injury (Figure 2(b)), while pretreatment with hypoxic CMECs-derived exosomes significantly attenuated these changes (Figure 2(b)). I/R injury increased the secretion of CK, LDH, IL-1*β*, and IL-18 (*p* < 0.01 vs. sham, Figure 2(c)). However, these changes were greatly prevented by intramyocardial injection of CMEC-derived exosomes, especially that from hypoxic CMECs. As for the effect of hypoxic exosomes on miRNAs, we found that the expression of miR-27b-3p, miR-17-1-2p, and miR-217-3p were downregulated in the periphery of the infarct zone after I/R injury (Figure 2(d)). However, the administration of CME-derived exosomes significantly reversed their expression (*p* < 0.05). As expected, the stimulation of hypoxic conditions was photographically confirmed by PCR analysis on the expression of miR-27b-3p, miR-17-1-2p, and miR-217-3p in CMECs (Figure 2(e)). miR-27b-3p expression was upregulated by hypoxia by 6-fold compared to normal condition (*p* < 0.0001); therefore, miR-27b-3p was selected to further study.

RETRACTED

### 3.3. Hypoxic CMEC-Derived Exosomes Protect H9C2 Cells against H/R Injury via miR-27b-3p

We found that the expression of miR-27b-3p in patients' plasma was significantly higher than that in normal people (Figure 3(a)). To confirm whether the effect of CMEC-derived exosomes on I/R injury was mediated by the upregulation of miR-27b-3p, the expression of miR-27b-3p was inhibited in CMECs. After transfection with miR-27b-3p inhibitor, the expression of miR-27b-3p was significantly inhibited in normal and hypoxic CMEC-derived exosomes (Figure 3(b)). In addition, the repair ability of hypoxic CMEC-derived exosomes on miR-27b-3p expression in the H9C2 H/R model was weakened by miR-27b-3p inhibitor compared to negative control (NC, *p* = 0.0138; Figure 3(c)). Immunofluorescence analysis showed the F-actin cytoskeleton was obviously reduced in H9C2 cells after H/R injury (Figure 3(d)). By contrast, the addition of CMEC-derived exosomes greatly upregulated F-actin expression, which was then downregulated by miR-27b-3p inhibitor (Figure 3(d)). The cellular uptake of PKH67-labeled exosomes into H9C2 cells was confirmed (Figure 3(d)), indicating that H9C2 cells successfully absorbed and integrated CMEC-derived exosomes.

We also confirmed that H/R injury significantly reduced the cell proliferation of H9C2 cells (*p* < 0.0001, Figure 3(g)). However, the addition of hypoxic CMEC-derived exosomes significantly rescued H/R injury-inhibited H9C2 cell proliferation. In comparison with exosomes with normal miR-27b-3p expression, those with inhibited miR-27b-3p expression had a significant lower effect on rescuing H9C2 cell proliferation from H/R injury (*p* = 0.0117, Figure 3(g)). Reverse results were found in the production of cellular LDH and cytokines (IL-1*β* and IL-18, Figure 3(e)). The productions of LDH, IL-1*β*, and IL-18 in H9C2 cell culture medium and the expressions of Foxo1, GSDMD, NLPR3, and caspase-1 proteins in H9C2 cells were significantly promoted by H/R injury (*p* < 0.0001, Figure 3(f)). Treatment with hypoxic CMEC-derived exosomes significantly reduced their elevation in the H9C2 H/R model. However, the inhibition of miR-27b-3p showed a weaker effect on reducing H/R-induced changes (*p* < 0.05, Figure 3(f)). By detecting the expression of oxidative stress-related factors of ROS and SOD in H9C2 cells after hypoxia-reoxygenation treatment, the results showed that hypoxia treatment induced the increase of ROS and the decrease of SOD secretion, CMEC-derived exosomes greatly upregulated ROS expression, which was then downregulated by miR-27b-3p inhibitor; however, the expression of extracellular SOD was the opposite (Figure 3(h)). These results indicated that miR-27b-3p played a role in promoting the protective effect of CMEC-derived exosomes against H/R injury.

RETRACTED

### 3.4. miR-27b-3p in Hypoxic CMEC-Derived Exosomes Attenuates H/R-Induced Injury and Pyroptosis in H9C2 Cells by Targeting Foxo1

We also found there were opposite expression pattern between miR-27b-3p and Foxo1 at the gene level (Figure 4(a)). The target pair between miR-27b-3p and Foxo1 gene was predicted using TargetScan database (Figure 4(b)) and then validated using the dual-Luciferase Reporter assay (Figure 4(c)). *In vitro* experiments were performed and H9C2 cells were treated with Foxo1 transfection, followed by transfection with miR-27b-3p inhibitor, H/R, and incubation with hypoxic CMEC-derived exosomes. The expression levels of miR-27b-3p and Foxo1 were found to be correlated in H9C2 cells. The expression of Foxo1 mRNA in the H9C2 H/R cell model was upregulated by the transfection with Foxo1 plasmid (*p* < 0.0001 for H/R+vector+NC-EXO versus H/R+Foxo1+NC-EXO, or H/R+vector+inhibitor-EXO versus H/R+Foxo1+inhibitor–EXO; Figure 4(d)), and this change was further enhanced by the miR-27b-3p inhibitor (*p* = 0.0003 for H/R+vector+inhibitor-EXO versus H/R+vector+NC-EXO, and *p* = 0.0002 for H/R+Foxo1+inhibitor-EXO versus H/R+Foxo1+NC-EXO). We observed a negative feedback loop between miR-27b-3p and Foxo1, as the expression of miR-27b-3p in H9C2 cells was downregulated by its inhibitors and Foxo1 overexpression (*p* < 0.01, Figure 4(e)).

Following Foxo1 overexpression, the expressions of F-actin and cell proliferation of H9C2 cells were inhibited (Figures 4(f) and 4(g)). The fluorescence intensity of F-actin protein and cell viability of H9C2 cells were reduced by Foxo1 expression (H/R+vector+NC-EXO>H/R+vector+inhibitor-EXO>H/R+Foxo1+NC-EXO>H/R+Foxo1+inhibitor-EXO). In addition, the expression of GSDMD, NLRP3, and caspase-1 proteins and the production of LDH, IL-1*β*, and IL-18 in H9C2 cells were increased accompanied with Foxo1 expression level (Figures 4(h) and 4(i)). These factors were increased by all treatments, especially by H/R+Foxo1+inhibitor-EXO. These results indicated that the overexpression of Foxo1 impaired the protective effect of hypoxic CMEC-derived exosomes in H9C2 cells and that the protective effects of miR-27b-3p in hypoxic CMEC-derived exosomes against H/R injury in H9C2 cells were mediated partially through decreasing Foxo1.

RETRACTED

### 3.5. Foxo1 Expression Impairs the Protective Effect of Hypoxic CMEC-Derived Exosomal miR-27b-3p against In Vivo I/R Injury and Promotes Pyroptosis

We first determined that the treatments with injection of lentiviral plasmid carrying Foxo1 and hypoxic CMEC-derived exosomes with the miR-27b-3p inhibitor obviously suppressed the protective effect of hypoxic CMEC-derived exosomes against I/R injury (Figure 5). The results showed that the expression of miR-27b-3p in the peri-infarct tissues in the rat heart was obviously decreased by injection of lentiviral plasmid carrying Foxo1 and hypoxic CMEC-derived exosomes transfected with miR-27b-3p inhibitors (Figure 5(a)). The expression level of miR-27b-3p in the rat heart was decreased sequentially from the greatest to the lowest by I/R+vector+NC-EXO, I/R+vector+inhibitor-EXO, I/R+Foxo1+NC-EXO, and I/R+Foxo1+inhibitor-EXO. After the I/R model was established, lentiviral plasmid expressing Foxo1 and exosomes (EXO) were injected into the rat heart. We found that the infarct area in rat hearts were increased by Foxo1 expression (*p* = 0.0302 between I/R+Foxo1+NC-EXO and I/R+vector+NC-EXO, and *p* < 0.01 between I/R+Foxo1+inhibitor-EXO and I/R+vector+inhibitor-EXO; Figure 5(b)). Lentiviral plasmid expressing Foxo 1 and exosomes (EXO) were injected into the rat heart, and then, the I/R model was established. The results showed that the ischemic areas in rat hearts were increased by Foxo1 expression (*p* = 0.0457 between Foxo1+I/R+NC-EXO and vector+I/R+NC-EXO, and *p* < 0.01 between Foxo1+I/R+inhibitor-EXO and vector+I/R+inhibitor-EXO; Figure 5(c)). The miR-27b-3p inhibitor in hypoxic CMEC-derived exosomes showed a significant contribution to ischemic areas (*p* = 0.153 between Foxo1+I/R+NC-EXO and Foxo1+I/R+inhibitor-EXO). HE staining of rat heart tissues indicated that pretreatment with Foxo1 plasmids counteracted the proactive effect of hypoxic CMEC-derived exosomes against fibrous hyperplasia, infiltration of inflammation cells, and increased disarrangement of myocardial cells (Figure 5(d)). Western blotting analysis showed that the expression of Foxo1, GSDMD, NLRP3, and caspase-1 proteins in peri-infarct tissues were increased by Foxo1 expression and miR-27b-3 inhibition (Figure 5(e)). The proportion of caspase-1-positive cells in the heart (Figure 5(f)) and the contents of serum CK, LDH, IL-1*β*, and IL-18 were increased in the same order (Figures 5(g) and 5(h)). The pretreatment with Foxo1 plasmids and miR-27b-3p inhibitor, especially the combined treatment of the two, significantly increased the production of pyroptosis-related proteins and serum CK, LDH, IL-1*β*, and IL-18. These results confirmed that the pretreatment with Foxo1 plasmids counteracted the proactive effect of hypoxic CMEC-derived exosomes against I/R injury in the rat model.

RETRACTED

### 3.6. Foxo1 Controls GSDMD Promoter Methylation and Histone Acetylation

Using MSP assay, we confirmed the transfection of miR-27b-3p mimics into H9C2 cells promoted methylation of the promoter region of the GSDMD gene, while the miR-27b-3p inhibitor reduced methylation level (Figure 6(a)). Next, the two binding sites of Foxo1 in the promoter region of GSDMD were predicted in JASPAR database (Figure 6(b)). Dual-Luciferase Reporter assay confirmed that the interaction between GSDMD promoter and Foxo1. We found the relative luciferase activities of dual-luciferase reporter carrying the wild-type binding sites of Foxo1 were greatly increased after the transfection of Foxo1 expressing plasmids (pcDNA-Foxo1, *p* < 0.0001, Figure 6(c)). No influence was found in the dual-luciferase reporters carrying the mutant binding sites of Foxo1. These results suggested the positive interaction between Foxo1 and GSDMD. ChIP-PCR showed that the expression of the GSDMD gene was downregulated in H9C2 cells treated with exosomes from hypoxic CMECs, whereas the inhibition of miR-27b-3p in hypoxic CEMCs partially rescued the expression of GSDMD (Figure 6(d)). The transfection with Foxo1 plasmids promoted relative higher level of H3K9AC antibody-captured DNA fragments of Foxo1 and decreased the level of HDAC2 antibody-captured DNA fragments (Figures 6(e) and 6(f)).

## 4. Discussion

Therapy methods using ECs, MSCs, and CPCs have made significant improvement in the treatment of I/R injury in preclinical experiments [11–16]. The underlying mechanism was associated with the alleviation of NLRP3 inflammasome-induced pyroptosis [16]. Inflammasome-induced pyroptosis after I/R injury could accelerate cardiac cell death, thereby aggravating I/R injury [9, 10]. Our present study analyzed the role of hypoxic CMECs-derived exosomesin myocardial regeneration after I/R injury, which were found to be associated with inflammasome-induced pyroptosis via miR-27b-3p-Foxo1 signaling.

RETRACTED

Hypoxia-elicited stem cell-derived exosomes show profound cardiac repair effect [31, 32]. In the damaged heart, exosomal miRNAs, especially those under hypoxia conditions, have demonstrated therapeutic values in several types of cells, including cardiomyocyte and CPCs [20, 22, 33]. Gray et al. showed the exosomes isolated from hypoxic CPCs improved tube formation ability of cardiac endothelial cells compared with exosomes derived from normal CPCs [22]. Moreover, they also identified that a cluster of miRNAs (miR-17, miR-103, and miR-15b) were upregulated in response to hypoxic conditions. miR-27b-3p is a tumor suppressor downregulated in several types of human cancers, including lung cancer [34], glioma [35], and breast cancer [36]. The feature of miR-27b-3p downregulation in patients with heart transplant rejection was previously identified [37]. The downregulation of miR-27b-3p in mouse cardiac fibroblasts was correlated with cardiac fibrosis [37]. At present, the relative expression of miR-27b-3p in cardiac endothelial cells and cardiomyocytes is still unclear. We demonstrated that the expression of miR-27b-3p in the rat heart was downregulated after I/R injury. The decreased expression of miR-27b-3p was associated with aggravated *in vitro* H/R injury of H9C2 cells and *in vivo* I/R injury of the rat heart.

Previous studies indicated the stimulation of hypoxia on a cluster of miRNAs and proteins with cytoprotection and proangiogenic effects [20, 22, 33]. miR-27b-3p exhibits various effects on drug metabolism, adipocyte differentiation, epididymal fat browning, acute kidney injury, and chemoresistance of tumor cells [38–41]. The fact that miR-27b-3p expression was upregulated in H9C2 cells under hypoxic conditions was in line with the results from previous studies [21–23, 25]. We determined that H9C2 cells *in vitro* or cardiomyocytes *in vivo* carrying hypoxic CMEC-derived exosomes had higher efficacy in alleviating I/R injury-induced inflammation, inflammation-mediated pyroptosis, and inhibition of cardiomyocyte proliferation when compared with exosomes derived from CMECs cultured under normal conditions.

Here, in our study, we confirmed that miR-27b-3p-mediated protective effect against I/R injury was mediated byFoxo1/GSDMD axis and NLRP3/caspase-1-induced pyroptotic cell death. NLRP3 inflammasome activation-mediated pyroptosis promotes myocardial I/R injury [10]. Huang et al. reported that emodin could reduce pyroptosis via suppressing the TLR4/MyD88/NF-*κ*B/NLRP3 inflammasome pathway, H/R-activated pyroptosis, and that NF-*κ*B or the NLRP3 inflammasome inhibitor reduced the expression of GSDMD-N and downregulated the expression of IL-1*β* [42]. Pyroptosis is mainly mediated by NLRP3 inflammasome-induced activation of caspase-1- and GSDMD-dependent secondary pyroptosis. Cellular damage, toxins, and infections can lead to the activation of inflammasome including Toll-like receptor 4 (TLR4) and NLRP3 [19], which recruit caspase-1 and then promote the production of pro-inflammatory cytokines such as IL-1*β* and IL-18 or activate GSDMD-mediated secondary pyroptosis [43–45] (Figure 7). Pyroptotic cells will subsequently release more inflammatory cytokines and toxins and stimulate the inflammatory and host defense responses and the injury [46]. Ge et al. demonstrated GSDMD-induced pyroptosis in myocardial I/R injury and that cardiomyocyte pyroptosis is mainly regulated via the caspase-11/GSDMD signaling pathway under oxidative stress conditions. Oxidative stress triggers GSDMD (gasdermin D) cleavage via CASP-11 (caspase-11). GSDMD-N oligomerizes and perforates the plasma membrane to mediate pyroptotic cell death. GSDMD, GSDMD-N, GSDMD-C, and IL- (interleukin-) 18 are released into the supernatant or peripheral blood. RIP3 refers to receptor-interacting protein 3 [47]. Xiang et al. suggested that mice with GSDMD knockout showed significantly reduce infarct size and improved cardiac function and postinfarction survival via reducing the release of IL-1*β* from neutrophil as well as the number of neutrophil and monocytes in infarcted hearts. It has been shown that GSDMD is necessary in improving the mobilization of neutrophil in infarcted hearts [48]. Our present study demonstrated the miR-27b-3p from hypoxic CMEC-derived exosomes attenuated IL-1*β* and IL-18, NLRP3, GSDMD, and caspase-1 induced by I/R injury, while the inhibition of miR-27b-3p impaired the mediated protective effects on the H9C2 cells and rat model. These results showed that miR-27b-3p exerted the cardioprotective effect partially through alleviating pyroptosis.

RETRACTED

Furthermore, miR-27b-3p-mediated cardioprotective and antipyroptosis effects were mediated by interacting with Foxo1 indirectly or directly promoting methylation of GSDMD promoter regions (Figure 7). Foxo1 acts as a transcription factor and has multiple functions through interacting with targets, including angiogenesis-related molecules [49]. Foxo1 could be influenced by various environmental stimuli including CK, oxidative stress, and hypoxia as well as various signaling such as Akt, NF-*κ*B, STAT3, and ERK1/2 [50–52] and is correlated with cellular behaviors including cell proliferation, differentiation, autophagy, cell cycle distribution, apoptosis, and DNA repair [53]. NLRP3 inflammasome-mediated pyroptosis was associated with Foxo1 [54, 55]. Foxo1-induced expression of NLRP3 inflammasome has been well confirmed in diabetes and insulin resistance [56, 57]. In addition, Foxo1 overactivation is reported to exacerbate myocardial I/R injury, whereas its downregulation contributes to the attenuation of myocardial I/R injury [58]. Our present study demonstrated that NLRP3-caspase-1 was activated by Foxo1 and miR-27b-3p. We also confirmed the binding of Foxo1 to GSDMD promoter, which indicated a positive regulation of Foxo1 on GSDMD-related pyroptosis (Figure 7). These results suggested that Foxo1 activation and miR-27b-3p inhibition could contribute to I/R injury and that the miR-27b-3p-Foxo1-mediated pyroptosis was of great significance in the progression of I/R injury. By contrast, the expression of miR-27b-3p was a protective factor against I/R injury.

I/R injury includes several types of cell death, such as necrosis, apoptosis, and iron ptosis. At present, we have only preliminarily studied the effect of pyroptosis; therefore, further experimental evidence is needed to prove that miR-27b-3p specifically inhibited focal death rather than other forms of cell death.

There were some limitations in this study. The exosomes derived from CMEC cells *in vitro* did not fully reflect the exocrine secretion of CMEC cells *in vivo*, and the treatment of I/R model rats with exosomes derived from CMEC cells also had some limitations. However, the current finding suggested that miR-27b-3p could be targeted in clinical therapy for patients with myocardial infarction or be used in early diagnosis by detecting miR-27b-3p expression in the serum of patients with myocardial infarction.

## 5. Conclusions

In summary, our present study indicated that hypoxia-induced expression of miR-27b-3p in CMEC-derived exosomes plays a crucial role in alleviating I/R injury via targeting Foxo1. Such an effect was mediated by GSDMD and NLRP3/caspase-1 mediated oxidative stress and pyroptosis. These results highlighted the potential of using hypoxic CMEC-derived exosomes for the treatment or prevention of I/R injury.

## Figures and Tables

**Figure 1:** The extraction and identification of exosomes. (a) The size of exosomes derived from CMECs in normal and hypoxic conditions. (b) The transmission electron microscopy (TEM) result for determining the exosomal morphology (scale bar = 100 nm). The figures are generated from NanoSight nanoparticle tracking analysis (NTA). (c) The expression of exosomal markers CD63, CD81, and TSG101 by Western blot analysis. EXO: exosomes.

RETRACTED

**Figure 2:** CMEC-derived exosomes prevent I/R injury and pyroptosis in the rat heart. Exosomes (EXO) were injected into the rat heart (intramyocardial injection). (a) TTC staining was used for the indication of the infarcted size in the rat heart. (b) The expression of Foxo1 protein and pyroptosis-related proteins in heart of rat with different treatments (*n* = 3). (c) The production of serum creatine kinase (CK), lactate dehydrogenase (LDH), interleukin- (IL-) 1*β*, and IL-18 by ELISA assay (*n* = 5). (d) The relative expression of miR-27b-3p, miR-17-1-2p, and miR-217-3p in heart of rat with different treatments (*n* = 5). (e) The relative expression of miR-27b-3p, miR-17-1-2p, and miR-217-3p in exosomes from CMECs cultured under normal and hypoxic conditions, respectively (*n* = 3). The sham group (*n* = 5), without ligation and reperfusion; the I/R group (*n* = 5), ischemia-reperfusion injury. The I/R+normal-EXO group (*n* = 5), exosomes, rats were administrated with exosomes (10 *μ*l, 6 × 10^12^ particles; intramyocardial injection) derived from CMECs cultured under normal conditions; the I/R+hypoxia-EXO group (*n* = 5), rats were administrated with exosomes (10 *μ*l, 6 × 10^12^ particles; intramyocardial injection) derived from CMECs cultured under hypoxic conditions.

**Figure 3:** miR-27b-3p is necessary for the cytoprotection of exosomes derived from CMECs in H9C2 cells. (a) The relative expression level of miR-27b-3p in patients and normal people (*n* = 16). (b) The relative expression level of miR-27b-3p in exosomes derived from CMECs cultured under hypoxic conditions with and without miRNA inhibitors (*n* = 3). (c) The relative expression level of miR-27b-3p in H9C2 cells with different treatments (*n* = 3). (d) Fluorescence analysis for the effect of the uptake of PKH67-labeled exosomes to the cytoskeleton of H9C2 cells. Scale bar = 20 *μ*m. (e) ELISA assay of the lactate dehydrogenase (LDH), interleukin- (IL-) 1*β*, and IL-18 in H9C2 cell culture medium (*n* = 3). (f) The expression of Foxo1 protein and pyroptosis-related proteins in H9C2 cells with different treatments. (g) Result of cell viability using CCK8 assay (*n* = 3). (h), the expression of ROS and SOD in H9C2 cells after different treatments. H/R: hypoxia/reoxygenation condition (2 h hypoxia: 5% CO_2_, and 95% N_2_; and 4 h normal conditions: 95% air plus 5% CO_2_). EXO: exosomes. NC-EXO or inhibitor-EXO indicated exosomes were derived from CMECs with pretreatment of negative control (NC) or miR-27b-3p inhibitor in hypoxic conditions.

RETRACTED

**Figure 4:** miR-27b-3p in hypoxic CMEC-derived exosomes attenuates H/R-induced injury and pyroptosis in H9C2 cells by targeting Foxo1. (a) The relative expression of Foxo1 in H9C2 cellular model under different treatments (*n* = 3). (b) The predictive targeting site of miR-27b-3p at the 3′UTR region of Foxo1 gene. Prediction was conducted in Targetscan Human database. (c) The Dual-Luciferase Reporter assay reported the interaction between Foxo1 and miR-27b-3p (*n* = 3). (d) The relative expression of Foxo1 in H9C2 cellular model in response to Foxo1 overexpression (*n* = 3). (e) Overexpression of Foxo1 decreased miR-27b-3p expression in the H9C2 H/R cell model (*n* = 3). This result shows a negative feedback between miR-27b-3p and Foxo1. (f) Overexpression of Foxo1 decreased the protective effects of exosomes on the cell viability of the H9C2 H/R cell model (*n* = 3). (g) Fluorescence analysis for the effect of the uptake of PKH67-labeled exosomes to the cytoskeleton of the H9C2 cell model with pretreatment of Foxo1 plasmids. Scale bar = 20 *μ*m. (h) Western blot analysis of the expression of Foxo1 protein and pyroptosis-related proteins. (i) Overexpression Foxo1 upregulated the production of lactate dehydrogenase (LDH), interleukin- (IL-) 1*β*, and IL-18 in the supernatant fluid of the H9C2 H/R cell model in response to exsomes (*n* = 3). H/R: hypoxia/reoxygenation (2 h hypoxia: 5% CO_2_ and 95% N_2_ and 4 h normal condition: 95% air plus 5% CO_2_). Caspase-1. EXO: exosomes. NC-EXO or inhibitor-EXO indicated exosomes were derived from CMECs with pretreatment of negative control (NC) or miR-27b-3p inhibitor in hypoxic conditions.

**Figure 5:** miR-27b-3p inhibition and Foxo1 expression show synergistically promotes I/R injury in rat heart. (a) The relative expression level of miR-27b-3p in peri-infarct heart tissues after I/R injury (*n* = 4). (b) The images and statistical results of infarcted sizes in rat heart (after the I/R model was established, lentiviral plasmid expressing Foxo 1 and exosomes (EXO) were injected into rat heart) (*n* = 4). (c) The images and statistical results of infarcted sizes in the rat heart (lentiviral plasmid expressing Foxo 1 and exosomes (EXO) were injected into rat heart; then, I/R model was established) (*n* = 5). (d) The representative images of histology (HE staining) of rat heart tissues (magnification, ×200, ×400; scale bar: 100, 50 *μ*m, respectively). (e) Western blot analysis of Foxo1 and pyroptosis-related proteins in the rat heart in response to different treatments. (f) The representative images of Foxo1 immunochemistry (magnification, ×200 and ×400; scale bar = 100 and 50 *μ*m, respectively). (g, h) The serum level of creatine kinase (CK), lactate dehydrogenase (LDH), interleukin- (IL-) 1*β*, and IL-18 in the rat heart (*n* = 5).

RETRACTED

**Figure 6:** miR-27b-3p controls the methylation of GSDMD promoter and Foxo1 promotes histone acetylation of GSDMD. (a) H9C2 cells were transfected with mi-27b-3p mimics or inhibiter; the methylation status of GSDMD promoter were detected by MSP. (b) The two predicted binding sites of Foxo1 in the promoter of the GSDMD gene. Their binding activity is predicted in JASPAR. (c) The Dual-Luciferase Reporter assay confirmed the interaction between Foxo1 and GSDMD at the two sites (*n* = 3). (d) The inhibition of miR-27b-3p in exosome derived from hypoxic CMECs increased the enrichment of GSDMD DNA (*n* = 3). (e, f) The ChiP-PCR results of GSDMD in 293 cells treated with Foxo1 expressing plasmids (*n* = 3).

**Figure 7:** The supposed schematic diagram of miR-27b-3p-Foxo1 mediated pyroptosis mechanism in I/R injury. Foxo1 expression on one hand induces GSDMD-mediated pyroptosis by activating the histone acetylation of GSDMD and, on the other hand, promotes NLRP3/caspase-1-mediated pyroptosis. Hypoxic CMECs-derived exosomes carrying high level of miR-27b-3p counteracted these interactions.

**Table 1:** The sequences of primers that were used in this study.

Name of gene	Primer	Sequence (5′-3′)
GAPDH	Forward	CCTCGTCTCATAGACAAGATGGT
	Reverse	GGGTAGAGTCATACTGGAACATG
U6	Forward	CTCGCTTCGGCAGCACA
	Reverse	AACGCTTCACGAATTTGCGT
All miRNA	Reverse	CTCAACTGGTGTCGTGGA
FOXO1	Forward	CAGCCAGGCACCTCATAACA
	Reverse	TCAAGCGGTTCATGGCAGAT
rno-miR-27b-3p	Reverse transcription	CTCAACTGGTGTCGTGGAGTCGGCAATTCAGTTGAGGCAGAACT
	Forward	ACACTCCAGCTGGGTTCACAGTGGCTAAGTT
rno-miR-17-1-3p	Reverse transcription	CTCAACTGGTGTCGTGGAGTCGGCAATTCAGTTGAGCCACAAGT
	Forward	ACACTCCAGCTGGGACTGCAGTGAAGGCACTT
rno-miR-217-5p	Reverse transcription	CTCAACTGGTGTCGTGGAGTCGGCAATTCAGTTGAGCCAGTCAG
	Forward	ACACTCCAGCTGGGTACTGCATCAGGAACTGA
Foxo1-GSDMD-ChIP	Forward	AGAGGCAGAGGCAGGTGAAT
	Reverse	GCCAATGGCTAAAGGACAAA
GSDMD (MSP)	M-F	TTCAGATCTTTTACTATGGCCCC
	M-R	CAGCCTGCCCTAGCCTTCTC
	U-F	TTTAGATTTTTTATTATGGTTTTGGTGT
	U-R	CAACCTACCCTAACCTTCTCCTC

## Data Availability

The data used in this research are available from the corresponding author on reasonable request.

## Supplementary Materials

Supplementary Materials Supplementary Figure 1: the identification of the isolated CMEC. The expression of CD31^+^ in isolated CMEC cells (magnification, ×200).
